The article "A meta-analysis of external fixator versus intramedullary nails for open tibial fracture fixation" was retracted in 2015. Reason: compromised peer review.

# A meta-analysis of external fixator versus intramedullary nails for open tibial fracture fixation

**DOI:** 10.1186/s13018-014-0075-6

**Published:** 2014-08-16

**Authors:** Xian Xu, Xu Li, Lin Liu, Wei Wu

**Affiliations:** 1 Department of Traumatic Orthopedics, East Hospital, No.150 Jimo Road, Pudong New District, Shanghai 200120, China

**Keywords:** Tibial fractures, Intramedullary nails, External fixator, Meta-analysis

## Abstract

**Background:**

To compare the clinical outcomes of external fixator (EF) and intramedullary nails (IN) in the treatment of open tibial fractures.

**Methods:**

We searched seven electronic databases (PubMed, MEDLINE, EMBASE, OVID, Cochrane library, CNKI, and CBM) for trials of tibial fracture fixation published from 1980 to 2013. The indicators including postoperative infection, malunion, nonunion, soft tissue injury, delayed healing, and healing time were used for quantitative outcome assessments.

**Results:**

A total of nine trials involving 532 patients (EF, *n* = 253; IN, *n* = 279) with open tibia fractures were included in this meta-analysis. The results indicated that the patients undergoing IN had lower incidence of postoperative infection (risk radio [RR] = 3.85; 95% confidence intervals [CI], 2.67–5.54; *P* < 0.0001), malunion (RR = 2.31; 95% CI, 1.40–3.81; *P* = 0.001), nonunion (RR = 1.41; 95% CI, 1.06–1.88; *P* = 0.02) and less healing time (weighted mean difference [WMD] = 6.19; 95% CI, 1.42–10.96; *P* = 0.01) compared with EF. However, regarding to the soft tissue injury (RR = 0.74; 95% CI, 0.34–1.62; *P* = 0.45) and delayed healing (RR = 1.38; 95% CI, 0.79–2.43; *P* = 0.26), there is no significantly difference between EF and IN approach.

**Conclusion:**

In conclusion, the use of IN is more effective than EF and may be considered as first-line approach in fixation of open tibial fractures.

## Introduction

Open tibial fractures are more frequent than any other long bone fractures, which are showing an increasing trend due to road traffic accidents and firearm injuries [1]. The management of open tibial fractures continues to be a major therapeutic problem because of the poor soft tissue cover and blood supply of the tibial shaft which make these fractures vulnerable to nonunion and infection [2]. Preventing tibia from postoperative infection, obtaining union, and returning the involved limb to normal function always remain elusive goals.

External fixator (EF) and intramedullary nailing (IN) are two common approaches for the fixation of open tibial fractures. Initially, the management by EF is well established as it allows immediate stabilization with access for management of the soft tissues [3],[4]. However, its use is also associated with significant rates of malunion and pin tract infection often necessitating premature removal and conversion to alternate forms of stabilization [5]-[7]. In addition, IN approach allows stable fixation with minimal additional violation of the soft tissues in the region of the fracture via placement of unreamed or reamed interlocking nails [8],[9]. The use of IN in treating open tibial shaft fractures results in a high rate of union and a low rate of infection and malunion [10]-[12]. Meanwhile, great benefits of EF for the fixation of open tibial fractures have been observed in shortening operation time, reducing blood loss and soft tissue injury, and improving blood supply at the broken ends of fractured bone and facture healing [13]-[16].

The article "A meta-analysis of external fixator versus intramedullary nails for open tibial fracture fixation" was retracted in 2015. Reason: compromised peer review.

Although EF and IN have been used as treatments of choice for tibial fractures, which of them can be served as an optimal approach still uncertain. There were some previous meta-analyses which supported the use of unreamed IN for open tibial fractures [17],[18]. However, the outcomes in recently published articles still remain controversy [19]-[21] and not all of them were included and reanalyzed in previous studies. Therefore, we conducted an updated meta-analysis with all the relevant studies to provide reliable evidence for the better efficacy of IN approach than EF in the fixation of open tibial fractures.

## Methods

### Search strategy

The literature search aimed to include all papers published between 1980 and 2013 that compared clinical outcomes of EF with IN approach in patients with open tibial fractures. The searched electronic database included PubMed, MEDLINE, EMBASE, OVID, Cochrane library, CNKI, and CBM.

All searches were carried out using the following keywords: ‘intramedullary nails’ , ‘external fixator’ , ‘tibia fractures’ , ‘fixation’ , and ‘tibia fractures’ , ‘external fixator’ , or ‘intramedullary nails’ and ‘tibia fractures’. The reference lists of any review papers and retrieved full-text manuscripts were scrutinized for additional articles.

### Eligibility criteria

Studies that met the following criteria were included in the meta-analysis: (i) they were randomized clinical trials (RCTs) or clinical controlled trials (CCTs), (ii) the participants were patients with open tibial fractures, and the diagnosis of tibial fractures was clearly defined, (iii) studies included the treatment of IN and EF, (iv) risk radio (RR) or weighted mean difference (WMD) as well as their 95% confidence intervals (95% CIs) were presented or the study provided enough data to calculate these values, (v) outcomes were accessed by at least one of the following indicators including postoperative infection, malunion, nonunion, soft tissue injury, delayed healing, and healing time, and (vi) the follow-up duration was more than 12 months.

The article "A meta-analysis of external fixator versus intramedullary nails for open tibial fracture fixation" was retracted in 2015. Reason: compromised peer review.

The studies should be excluded if they were (i) case-based reports, (ii) publications of surgical protocols or technical manuals, (iii) studies with lack of access to the full text, (iv) studies related to closed tibia fractures, and (v) duplicated publications.

### Data extraction

Data was extracted independently by two reviewers (Wei Wu and Lin Liu) using a predesigned data extraction form. The detailed data including title, year of publication, sample size, gender and age of participants, types of tibia fractures, design of study (RCT or CCT), blinding, materials of fixation, number of patients who dropped out, and outcomes were recorded. Any disagreements were resolved by discussion with the colleagues (Xian Xu and Xu Li).

### Outcome measures

In the meta-analysis, the indicators including postoperative infection, malunion, nonunion, soft tissue injury, delayed healing, and healing time were used for quantitative outcome assessments.

### Methodological quality

The methodological quality of included trials was assessed by using the Jadad score [22], which is a validated five-point scale (0–2, poor quality; 3–4, good quality; 5, excellent quality) that examines the methods of randomization, double-blinding, and the reporting of withdrawals and dropouts. One point was given when one of the following five criterions was met: (1) randomized study, (2) randomization described, (3) double-blind study, (4) double-blinding described, and (5) description of withdrawals and dropouts.

### Statistical analysis

One author (Xian Xu) conducted all statistical analyses using Review Manager 5.0 provided by the Cochrance Collaboration. Dichotomous data results (postoperative infection, malunion, nonunion, soft tissue injury, and delayed healing) were summarized using RR and 95% CIs. Continuous outcomes (healing time) were summarized by the WMD and 95% CIs. The heterogeneity among studies was accessed by Chi-square test of Q and *I*^2^ statistics with significance set at *P* < 0.05 and *I*^2^ > 50% [23]. When no significant heterogeneity was found, a fixed effect model was used to pool the data. Otherwise, we used a random effect model. The significance of the pooled RR or WMD was determined by the *Z*-test, and *P* value < 0.05 was considered statistically significant.

## Results

### Study characteristics

In the initial literature search on the electronic database, a total of 628 citations were identified. After removing the duplicated articles, 336 literatures were remained. Then, 271 obvious irrelevant articles were excluded. Among the remaining 65 articles, there were 5 animal studies, 34 noncontrolled or non-RCT trials, 6 cases of closed tibia fractures, 1 case of tibia fracture in children, 9 literature reviews, and 1 repeatedly published paper. After excluding them, nine papers met the inclusion and exclusion criteria (Figure 1).

The article "A meta-analysis of external fixator versus intramedullary nails for open tibial fracture fixation" was retracted in 2015. Reason: compromised peer review.

**Figure 1:** Literature search and study selection.

Finally, nine randomized trials were identified to do this meta-analysis [19]-[21],[24]-[29]. The included studies were published during the period 1989–2011. Table 1 summarizes the characteristics of these studies including research time, facture types, sample size, gender and age of participants, and materials for fixation. In total, 532 patients aged 28–87 years were treated with EF (*n* = 253) or IN (*n* = 279). Fractures in all selected trials were diagnosed as Gustilo-Anderson type II or III [30] except the study of Holbrook et al. [29]. In addition, the Jadad quality score of each included studies is shown in Table 2. All the studies were randomized studies and described the randomization. No studies used double-blind method and described the withdrawals and dropouts.

**Table 1:** Characteristics of selected trials

**Author published year**	**Time of research**	**Study design**	**Types of fractures**	**Number**		**Materials**		**Gender (F/M)**		**Age**	
				**EF**	**IN**	**EF**	**IN**	**EF**	**IN**	**EF**	**IN**
Antrich-Adrover [26] 1997	NA	RCT	II/IIIA/B	22	17	NA	NA	19/3	11/6	29.7 ± 19.4	32.6 ± 15.7
Cozma [24] 2000	1994.1–1998.12	CCT	IIIA/B/C	29	33	Burghele/Ilizarov	Unreamed	36/21		36 (17–70)	
Henley [25] 1998	1988.1–1993.3	CCT	II/IIIA/B	68	100	Half-pin	Unreamed	53/15	79/21	33 (16–77)	33 (14–81)
Inan [19] 2007	1997.3–2000.5	RCT	IIIA	32	29	Ilizarov	Unreamed	28/4	24/5	32.3 (15–64)	31.7 (17–54)
Mohseni [20] 2011	2009.3–2011.3	RCT	IIIA/B	25	25	AO tubular plate	Unreamed	22/3	20/5	28.92 ± 8.88 (12–49)	30.8 ± 5.24 (23–39)
Shannon [21] 2002	NA	RCT	IIIA	17	13	AO tubular plate	Unreamed	10/7	7/6	34 (17–71)	44 (21–82)
Tornetta [27] 1994	1989.1–1991.1	CCT	IIIB	14	15	NA	NA	9/5	11/4	37 (19–86)	41 (21–73)
Tu [28] 1995	1992.1–1992.6	RCT	IIIA/B	18	18	Hoffmann	NA	30/6		38.5 (16–85)	
Holbrook [29] 1989	1985.7–1987.9	RCT	I/II/III	28	29	AO/Hoffmann/Orthofix	NA	NA		25 (7–65)	28 (15–66)

*EF* external fixation, *IN* intramedullary nails, *NA* not provided.

**Table 2:** Jada quality score of randomized, controlled trials included in the meta-analysis

**Reference**	**Randomization**	**Double blinding**	**Withdrawals and dropout**	**Total score**
Antrich-Adrover [26]	2	0	0	2
Cozma [24]	2	0	0	2
Henley [25]	2	0	0	2
Inan [19]	2	0	0	2
Mohseni [20]	2	0	0	2
Shannon [21]	2	0	0	2
Tornetta [27]	2	0	0	2
Tu [28]	2	0	0	2
Holbrook [29]	2	0	0	2

The article "A meta-analysis of external fixator versus intramedullary nails for open tibial fracture fixation" was retracted in 2015. Reason: compromised peer review.

### Postoperative infection

The incidence of postoperative infection was reported in 7 out of 9 included studies [19]-[21],[24],[25],[28],[29] including 471 patients (EF, *n* = 220; IN, *n* = 251). The heterogeneity among studies was not significant (*P* = 0.12, *I*^2^ = 40%), so the fixed-effect model was used to pool the data. The results (RR = 3.85; 95% CI, 2.67–5.54; *P* < 0.0001) indicated that the incidence of postoperative infection in patients treated with EF approach was significantly higher than that in patients treated with IN approach (Figure 2A).

**Figure 2:** **Forest plots for comparing the clinical outcomes between intramedullary nails and external fixation. (A)** Postoperative infection. **(B)** Malunion. **(C)** Nonunion. **(D)** Soft tissue injury. **(E)** Delayed healing. **(F)** healing time.

### Malunion

Seven trials [19],[20],[24],[26],[28],[29] with 334 patients (EF, *n* = 168; IN, *n* = 166) investigated the occurrence rate of malunion in patients treated with EF or IN approach. No significant heterogeneity was observed between these studies (*P* = 0.56, *I*^2^ = 0%), and fixed effect model was used. The overall RR of malunion was 2.31 (95% CI, 1.40–3.81; *P* = 0.001), indicating that occurrence rate of malunion was significantly lower in patients undergoing IN compared with EF (Figure 2B).

### Nonunion

Clinical outcome of nonunion was evaluated in seven trials [19]-[21],[24],[26],[28],[29], including 447 participants (EF, *n* = 212; IN, *n* = 235). No significant heterogeneity was existed in the included studies (*P* = 0.55, *I*^2^ = 0%). Thus, the fixed effect model was applied for pooling data. The summary RR for disunion was 1.41 (95% CI, 1.06–1.88; *P* = 0.02), indicating that the incidence of disunion was reduced by IN compared with EF (Figure 2C).

### Soft tissue injury

Two included studies [20],[21] containing 80 patients (EF, *n* = 38; IN, *n* = 42) reported the soft tissue injury of the patients treated with EF or IN approach. There was no significant heterogeneity between the two studies (*P* = 0.29, *I*^2^ = 10%), so a fixed effect model was adopted. The pooled estimate (RR = 0.74; 95% CI, 0.34–1.62; *P* = 0.45) showed that there was no significant difference in soft tissue injury between EF and IN approach for the patients with open tibia fractures (Figure 2D).

### Delayed healing

Three trials [19],[25],[29] including 292 patients (EF, *n* = 130; IN, *n* = 162) evaluated the delayed healing of EF and IN for open tibia fractures patients. Due to no significant heterogeneity among studies (*P* = 0.96, *I*^2^ = 0%), fixed-effect model was adopt. No significant difference in delayed healing was identified between the patients treated with EF and IN approach (RR = 1.38; 95% CI, 0.79–2.43; *P* = 0.26) (Figure 2E).

The article "A meta-analysis of external fixator versus intramedullary nails for open tibial fracture fixation" was retracted in 2015. Reason: compromised peer review.

### Healing time

The healing time was reported in three included studies [21],[26],[29] with 261 patients (EF, *n* = 115; IN, *n* = 146). Significant heterogeneity was existed in the studies, so random effect model was used (*P* = 0.04, *I*^2^ = 70%). The overall estimate (WMD = 6.19; 95% CI, 1.42–10.96; *P* = 0.01) indicated that the healing time was significantly reduced by IN approach compared with EF (Figure 2F).

## Discussion

### Main findings

IN and EF are two common approaches for the fixation of tibial fractures. In this study, we compared the efficacy of them for open tibial fractures. The results indicated that the patients undergoing IN had lower incidence of postoperative infection, malunion, nonunion, and less healing time compared with EF [25]. However, regarding to the soft tissue injury and delayed healing, there was no significantly difference between EF and IN approach. This may be explained, at least in part, by the short number of studies that evaluated the clinical outcomes of soft tissue injury and delayed healing.

The result of this study was consistent with the previous meta-analyses [17],[18]. Compared with them, the study published in 2002 [21] was included in this study, which was not analyzed in the previous meta-analyses. In addition, the indicators of soft tissue injury, delayed healing, and healing time were used to compare the efficacy of EF and IN in this study. The superior of IN was more comprehensively proved by this meta-analysis.

### Clinical implications

The results of this study should be of value not only to clinicians considering EF versus IN therapy for their patients with open tibia fractures but also for researchers in the field of osteology. For the most clinical endpoints studied in this meta-analysis, IN group has considerably higher efficacy for treatment of open tibia fractures compared to EF. However, the efficacy of IN would vary according to different materials of nails including unreamed and reamed nails. The unreamed technique can offer stability and anatomic alignment of the affected bone, even in the presence of bone loss or comminution [27],[31]. Conversely, a previous meta-analysis reported by Duan et al. has indicated that reamed intramedullary nailing has better treatment effects than unreamed intramedullary nailing for shaft fracture of femur in adults, with significant lower reoperation rate, lower nonunion rate, and lower delay union rate [32]. In this meta-analysis, four trials [26]-[29] did not report the important data of nail types that were used for the fixation of tibial fractures. Therefore, further investigations are required to improve understanding of differences between different types of intramedullary nails and external fixation.

The article "A meta-analysis of external fixator versus intramedullary nails for open tibial fracture fixation" was retracted in 2015. Reason: compromised peer review.

### Limitations

Some limitations of this study should be acknowledged. First, the significant heterogeneity was found among the studies in the analysis of healing time. No analysis for exploring heterogeneity sources was performed in this study due to lack of enough data. Thus, further studies must be done to explore the heterogeneity sources. Second, because the recruited studies were not double blind, and incidence of withdrawals and dropout were not mentioned (total Jadad score = 2), there is still a need for more and higher quality case-control studies to test and verify the results of this meta-analysis. Third, funnel plot as a tool for detection of selection-related biases should be applied in this meta-analysis.

## Conclusion

IN approach may improve postoperative outcomes such as postoperative infection, malunion, disunion, and healing time; thus, it may be used as a first-line treatment for patients with open tibial fractures.

## Abbreviations

EF: external fixator

IN: intramedullary nails

RCT: randomized clinical trial

CCT: clinical controlled trial

RR: relative risks

OR: odds ratios

SMD: standardized mean difference

## Competing interests

The authors declare that they have no competing interests.

## Authors’ contributions

XX and XL conceived of the study and participated in its design and coordination. LL designed and performed the experiments, and collected the data. WW wrote the manuscript. All authors read and approved the final manuscript.
